RETRACTED

# Analysis of Multiple Human Tumor Cases Reveals the Carcinogenic Effects of PKP3

**DOI:** 10.1155/2021/9391104

**Published:** 2021-10-25

**Authors:** Shujie Ruan, Jingping Shi, Ming Wang, Zhechen Zhu

**Affiliations:** The First Affiliated Hospital with Nanjing Medical University, Jiangsu Province Hospital, Nanjing 210029, China

## Abstract

Plakophilins (PKPs) act as a key regulator of different signaling programs and control a variety of cellular processes ranging from transcription, protein synthesis, growth, proliferation, and tumor development. The function and possible mechanism of PKP3 in ovarian cancer (OC) remain unknown. It is extremely important to investigate the expression and prognostic values of PKP3, as well as their possible mechanisms, and immune infiltration in OC. Therefore, in this paper we explored the potential oncogenic role of PKP3 in 33 tumors based on The Cancer Genome Atlas (TCGA) and Gene Expression Omnibus (GEO) datasets. The result outcomes showed that PKP3 is highly expressed in most cancers, and the expression level and prognosis of PKP3 showed little significance in cancer patients. Moreover, oncologists have found that members of the plakophilin family have different degrees of abnormality in ovarian cancer. PKP3 played a key part in carcinogenesis and aggressiveness of OC as well as malignant biological activity and can be used as a biomarker for early diagnosis and prognosis evaluation in OC.

## 1. Introduction

Cancer is the next leading cause of mortality in the globe, claiming the lives of more than 8 million people each year. Tumors are classified as cancers because they are caused by the growth and spread of somatic cell clones that are self-expanding [1, 2]. If the cancer clone is going to behave in this way, it will have to co-opt multiple cellular pathways that allow it to ignore normal cell growth constraints, modify the local microenvironment to favor its proliferation, infiltrate through tissue barriers, spread to other organs, and escape immune surveillance [3–5]. Because carcinogenesis is complicated, it is necessary to do a pan-cancer expression study of an intriguing gene and analyze its association with clinical prognosis and probable molecular processes. Functional genomics datasets, such as the TCGA project and the GEO database, allow us to analyze any target gene in depth [6–10]. PKPs regulate a range of cellular activities, including RNA transcription, protein synthesis, proliferation, tumor growth, and destiny determination [11].

Desmosome-bearing cells, except for hepatocytes and cardiomyocytes, may be targeted with great specificity by PKP3. They observed that loss of PKP3 leads to a reduction in desmosome size, as well as an increase in cancer migration [12–17]. The eight ARM repeat domains (ARM1–8) were discovered in the human PKP3 protein. According to new findings from a variety of studies, PKP3 has functional connections with anomalies in the hair follicle system as well as with skin inflammation responses and carcinogenesis. Recent cell or animal-based research shows that PKP3 has a role in carcinogenesis and development. Current cancer research has not thoroughly clarified the link between PKP3 and various cancers, which is based on extensive clinical data [18, 19]. As a result of our analysis and discussion of PKP3, we have discovered that it may be an important therapeutic target in different cancers and that PKP3 may play an important role both during the pathogenesis of cancer and in the clinical prognosis of cancer. We hope that our work will help to fill this knowledge gap. The framework of the proposed model is depicted in Figure 1.

RETRACTED

The rest of the paper is organized as follows. In Section 2, the proposed system model's materials and methods are described. The experimental results are further summarized in Section 3.  Section 4 provides detail discussion on results. Finally, Section 5 concludes the paper with summary and future research directions.

## 2. Materials and Methods

### 2.1. Benchmark Dataset

We collected genome data from the Genomic Data Commons (GDC) data portal website, namely 33 tumor patients' tumor RNA-seq data, comprising mRNA expression data and miRNA expression data [20–22]. Each tumor is matched with a normal tissue sample. Based on the downloaded data, we split the dataset into two groups [23, 24] and labeled them tumor samples and normal tissue samples, respectively. During the study, we set the *p* value cutoff to 0.01, the log2 (fold change) cutoff to 1, and we utilized the R program to create the PKP3 heat map [25]. Furthermore, all TCGA tumors were simply divided into four stages based on their pathological stages (stage I, stage II, stage III, and stage IV), and the violin diagrams of PKP3 expression in different pathological stages of different tumors were analyzed and plotted based on the analysis modules we had accumulated [14]. In this study, the expression data from the log2 transformation are utilized for either the box or the violin diagram. According to reports, the UALCAN tool is an interactive Web resource for analyzing cancer omics data. UALCAN was utilized in this work to examine and analyze PKP3 protein expression levels, and the particular operational procedures were done step by step according to the instructions provided on the Web page.

Moreover, we did not investigate the protein expression level of PKP3 in the remaining malignancies in this investigation due to a lack of proteomic data except for breast cancer, ovarian cancer, colon cancer, renal cell carcinoma (clear cell RCC), uterine corpus endometrial carcinoma (UCEC), and lung adenocarcinoma (LUAD).

RETRACTED

### 2.2. Survival Prognosis Analysis

The survival module of the GEPIA2 online open tool was used in this study to obtain the overall survival (OS) and disease-free survival (DFS) significance map data for PKP3 in all 33 tumors within the TCGA project. According to the high (50%) and low (50%) cutoff values as the criteria of high and low expression threshold, the data were separated into high-expression and low-expression cohorts. The log-rank test was used for hypothesis testing, and the GEPIA2 tool was also used in this study to obtain survival graphs. We also detected the survival prognosis of all tumors by the ACLBI Web tool [26–28]. Opening the website, we input “PKP3” in the prognosis module after we selected the TCGA cancer type and then had got the survival prognosis analysis results of PKP3 in the corresponding cancer cases. All analysis operations were performed using open source tools on the Web and in accordance with the instruction manual.

### 2.3. Genetic Alteration Analysis in 33 Tumors

Because there is no corresponding gene mutation analysis package and ready-made process in our R language package, we found the cBioPortal website (https://www.cbioportal.org/) reported in the literature to summarize the mutations occurring in the genome [29–32]. First of all, we created a new account to log in cBioPortal; then we found the search box in the module of TCGA Pan-Cancer Atlas Studies and input PKP3 to query the genetic alteration characteristics of PKP3 in 33 tumors. In the “Cancer Type Summary” module, we obtained the change frequency of PKP3, type of mutation, and copy number alteration (CNA) in all tumors. The “Mutations” module shows a three-dimensional protein structure of the mutation site based on previous research information. To better understand the differences in survival due to PKP3 mutations, we obtained and analyzed data on overall, disease-free, progression-free, and disease-free survival differences in 33 cancer cases with or without PKP3 mutations [33]. Kaplan–Meier plots with log-rank *p* values were generated as well. In contrast to the genetic alteration analysis, we detected and summarized the phosphorylation sites and levels of PKP3 protein in the UniProt website.

### 2.4. Immune Cell Infiltration Analysis in TCGA Project

Immune cell infiltration has been reported to be an important factor leading to changes in the microenvironment of tumor cells. Therefore, in this study, the relationship between PKP3 expression and immune cell infiltration was analyzed in detail. The Timer2 Web server was employed in this work to perform the analysis. The immune cells of cancer-associated fibroblast cells, B cells, T follicular helper cells, and Treg cells were selected in this part. For reliable immune score evaluation, we used an R software package that integrates six latest algorithms, including TIMER [22], xCell [34], MCP-counter, CIBERSORT, EPIC, and quanTIseq [27, 28, 35], to do detect the immune score. The *p* values and partial correlation (COR) values were obtained via the purity-adjusted Spearman's rank correlation test and the rank sum test. Those above data were summarized and visualized as a heat map and a scatter plot within R packages.

RETRACTED

### 2.5. PKP3-Related Gene Enrichment Analysis

We queried the functional network of PKP3 in the STRING website using protein names and biological organisms as constraints [36]. And, in the analysis, major parameters such as minimum interaction score, network edge, maximum number of interactive users to be displayed, and active interaction sources are set as “low confidence (0.15),” “evidence,” “no more than 200 interactive users,” and “experiments,” respectively. Finally, after several parameter adjustment attempts, we successfully obtained an available determined PKP3 binding protein dataset. In addition, the GEPIA2 “Similar Gene Detection” module, based on the dataset of all TCGA tumors and normal tissues, was used to obtain the top 200 targeting genes associated with PKP3 [24]. Pairwise gene association analysis was performed on PKP3 and the selected genes using the Pearson correlation analysis method, and the analysis results were visualized into a dot plot (the log2 TPM), and the *p* value and the corresponding correlation coefficient (*R*) were calculated. In addition, the heat map data of selected genes containing partial correlation (COR) and *p* values in Spearman's rank correlation test after purity adjustment were evaluated by using the “Gene_Corr” module of TIMER2. Genetic analysis of PKP3 binding and interaction was performed using the interactive Venn diagram viewer jvenn for cross analysis. Finally, we combined the two sets of data to perform KEGG (Kyoto Encyclopedia of Genes and Genomes) pathway analysis. All analysis results are visualized by the R language software package and tested by the two-tailed hypothesis test.

## 3. Experimental Results

### 3.1. PKP3 Differentially Expressed in Tumors

The pan-cancer analysis is acknowledged as a strong method for analyzing the involvement of target genes in different malignancies [25]. We used public datasets and advanced analysis technologies to investigate the function of PKP3 in different tumor types. PKP3's protein structure (NM 001303029.2 for the mRNA or NP 001289958.1 for the protein) is conserved among diverse species including humans, musculus, and *B. taurus* (ARM1–8). We used public datasets and advanced analysis technologies to investigate the function of PKP3 in different tumor types. In Figure 2, PKP3's protein structure (NM 001303029.2 for the mRNA or NP 001289958.1 for the protein) is conserved among diverse species including humans, musculus, and *B. taurus* (ARM1–8). Molecular evolutionary genetic analysis was used to determine the evolutionary relationship of PKP3 among different species. The evolutionary relationship was then displayed as part of the phylogenetic tree. According to these findings, PKP3 is functionally and physically conserved across a wide range of species. There are substantial differences in how PKP3 is expressed in different organs. Our study revealed that when comparing the HPA (human protein map), GTEX, and FANTOM5 datasets, PKP3 protein expression is greatest in the skin. It was revealed in the NCBI database; however, the PKP3 mRNA was expressed in up to 15 tissues, which indicates a high degree of tissue specificity. Researchers have determined that the physiological threshold concentration of PKP3 in cells is around 2.9 g/L, according to proteomics and mass spectrometry data.

RETRACTED

When it comes to tumor cells, however, PKP3 expression has not been thoroughly studied. PKP3 expression levels were measured in 33 cancers using Timer2. A greater expression of PKP3 was found in the tumor tissues compared with the equivalent control tissues (Figure 2(a)). Due to the lack of PKP3 expression information in several normal tissues, we further analyzed the differences in PKP3 expression levels between tumor tissues and adjacent normal tissues in the GTX database. Based on PKP3 expression information from the two databases, however, no difference in PKP3 expression was observed in adrenocortical carcinoma (ACC), lymphoid neoplasm diffuse large B-cell lymphoma (DLBC), and mesothelioma (MESO) tissues compared with normal tissues. These results suggest that PKP3 may play a different role in different tumors. We next used the CPTAC dataset to investigate the expression levels of total PKP3 protein in the primary tissues of six different tumors, including breast cancer, colon cancer, clear cell RCC, LUAD, UCEC, and OV.

The total protein expression was greater in primary tissues of breast cancer, colon cancer, clear cell RCC, LUAD, UCEC, and OV than in normal tissues, as shown in Figure 3(a). These findings are congruent with the published publications and summary analysis results in the Oncomine database, indicating that our findings are very trustworthy. In addition, we performed pathological staging on 33 tumors and discovered a link between PKP3 expression and tumor pathological stages to develop markers for therapy or determine various tumor stages (Figure 3(b)).

RETRACTED

### 3.2. PKP3 Expression Difference and Survival Prognosis

According to the expression level of PKP3, tumor cases were separated into high-expression and low-expression groups and the association between PKP3 expression and prognosis of various tumor patients was investigated using the TCGA and GEO datasets, respectively. High PKP3 expression in the TCGA program was linked with poor overall survival (OS) for CESC, Kirc, LiHC, MESO, PAAD, and SKCM malignancies, as shown in Figure 4(a). Data from the disease-free survival (DFS) study revealed that low PKP3 expression was inversely associated with a better prognosis in KIRC, LUSC, MESO, PAAD, and PRAD. Furthermore, Kaplan–Meier survival data analysis revealed that decreased PKP3 expression was linked with a worse OS and progression-free survival (PFS) prognosis in ovarian cancer (OV). High PKP3 expression was associated with a worse overall survival (OS), postprogressive survival (PPS), and first progressive (FP) prognosis in patients with lung cancer (LC) (Figure 4(b)) and a worse disease-specific survival (DSS) prognosis in patients with liver cancer (LIC). Furthermore, increased PKP3 expression was associated with a poor prognosis of OS, FP, and PPS in gastric cancer (GC). Our analytical data confirmed that PKP3 expression was associated with prognosis in ovarian, lung, and gastric cancers, but not in breast cancers. These data suggest that the expression of PKP3 differs from the prognosis of patients with different tumors.

### 3.3. Mutated PKP3 Correlated with Survival Prognosis

In this section, Figure 4(a) shows that the largest modification frequency (>4.5%) of PKP3 occurs in individuals with brain lower grade glioma tumors that have “deep deletion” as the main type. In skin-cutaneous melanoma instances, the “mutation” form of CNA predominates, with an alteration frequency of 4 percent. And in diffuse large B-cell lymphoma, the “fusion” form accounted for 2 percent of the disease (Figure 5(a)). As a sidenote, PKP3 has genetically altered in all cases of testicular germ-cell cancer as well as adrenocortical cancer and esophageal adenocarcinoma tumors (Figure 4(a)). Figure 4(b) further shows the type, location, and number of cases of the PKP3 gene mutation. We found that missense mutation is the main type of PKP3 genetic modification. The S323L/P change in the arm repeats is detected in 2 cases of cervical squamous cell carcinoma and 1 case of gastric tubular adenocarcinoma (Figure 5(b)) and transforms the PKP3 protein from serine (S) to leucine (L) or proline (L) at site 323. The L323 and L464 sites' alteration of PKP3 was shown in the 3D structure in Figure 4(c).

RETRACTED

We also explored the potential relationship between PKP3 mutation and the clinical survival prognosis of patients with different types of cancer. We further compared the overall survival, progression-free survival, disease-specific survival, and disease-free survival prognosis of tumor patients with PKP3 mutations. Compared with cases with unmutated PKP3, the data in Figure 6 show that BLCA but no other cancer cases carrying mutations in PKP3 showed poorer overall survival prognosis, rather than disease-specific survival, disease-free survival, and progression-free survival prognosis.

### 3.4. Methylation of PKP3 DNA in Tumorigenesis

Since DNA methylation levels and cancer and development are both strongly connected, the MEXPRESS technique was utilized to explore the possible relationship between DNA methylation levels and tumorigenesis and survival prognosis of various malignancies. To our surprise, we found substantial DNA methylation at several promoters and nonpromoter probes, such as those for cg10112265, cg06144018 cg06267084, or 24982763 in instances of BLCA tumors but not GBM tumors (Figure 7). Also using UALCAN, researchers analyzed PKP3 gene methylation in BLCA tissues (*n* = 418) and normal tissues (*n* = 21) at different stages, with or without mutations in TP53.

Based on methylation data, we detect differences between the normalized data and that of the normal tissues and the BLCA tissues (Figures 8(a)–8(f)). Unfortunately, we did not examine the link between DNA modification and the level of PKP3 expression in our study due to a lack of data. So far, no research has looked at whether the nonpromoter methylation of the PKP3 gene impacts the production or homeostasis of PKP3 protein. In future publications, we will continue to explore PKP3 using the big data platform.

### 3.5. Multisite Phosphorylation Modification in Tumor Tissues

For this study, we looked at the differences between normal and primary tumor tissues in terms of the expression levels of PKP3. Breast cancer, clear cell RCC, LUAD, and UCEC tumors were selected as representative tumors in this study. Amino acid alteration locations and substantial changes are summarized in Figure 9(a). A nice surprise is that all the primary tumor tissues (Figures 9(b)–9(e)) had greater phosphorylation of the ARM repeat domain of PKP3 than normal tissues, but not the serine or threonine, which is commonly phosphorylated in proteins. We only looked at the PKP3 phosphorylation levels in normal tissues, and as indicated, we discovered elevated phosphorylation of S331, S314, T250, S240, S238, and S183, the regions inside the ARM repeat domain. This finding warrants additional investigation into the potential involvement of S138, S145, S211, and S329 phosphorylation in carcinogenesis.

RETRACTED

### 3.6. PKP3 Associated with Multiple Immune Cell Infiltration

Tumor-infiltrating immune cells are considered to be a prominent factor of regulating tumor microenvironment homeostasis and regulating the tumorigenesis, progression, or metastasis of cancer. Those cells in the tumor matrix have been reported to participate in the regulation of cancer progression. Therefore, multiple algorithms such as TIMER, CIBERSORT-ABS, CIBERSORT, MCP-counter, QUANTISEQ, XCELL, and EPIC are used to study the potential relationship between different immune cells (NK cells, B cells, T cells, macrophages, etc.) and PKP3 gene expression in diverse cancer types of TCGA projects. After analyses, we observed a statistical lower immune infiltration of B cells, T cells, and macrophages in the tumors of LUSC and TGCT metastasis based on most algorithms (Figures 9 and 10). We further studied the infiltration of immune cells was involved in the cancer through the analysis of TCGA projects in detail. In addition, the analysis results showed a positive correlation between PKP3 expression and CD8^+^ T-cell infiltration in the ACC tumor microenvironment (Figures 10(a)–10(c) and 10(f)) and a negative correlation between PKP3 expression and CD8^+^ T-cell immune infiltration in PAAD from Figures S8(a)–S8(c).

As shown in Figures 10(a)–10(c), we were surprised to find that PKP3 expression was positively correlated with the estimated infiltration of cancer-associated fibroblasts in the ACC tumors. And we also got a positive correlation between the Treg cell and T follicular helper cell infiltration and PKP3 expression in the tumors of BRCA from Figures 10(b)-10(c). In order to further confirm the correlation between PKP3 expression and the infiltration of immune cells, we used the CIBERSORT-ABS algorithm in the software to calculate the infiltration levels of various immune cells. The scatter plot data are presented in Figures 10(d)–10(f). It is obvious that the PKP3 expression level in BLCA, BRCA, and LGG is positively correlated with the infiltration of T follicular helper cells. To sum up, PKP3 is associated with a variety of immune cell infiltrates, and these results suggest that PKP3 may be a novel therapeutic target for different types of tumors and should be taken into account when treating.

RETRACTED

### 3.7. Enrichment Analysis of PKP3-Related Partners

Study results show that PKP3 can cause carcinogenesis and alter survival prognoses as well as alter the tumor microenvironment. So that we could study the PKP3 mechanism in depth; we tried to filter out proteins that associate with PKP3 and genes linked to PKP3. A successful STRING tool search yielded 200 experimentally validated protein-PKP3 binding proteins. This is accomplished in two ways. First, using the STRING tool, we successfully identified 200 experimentally confirmed proteins that interact with PKP3 (Figure 11(a)). Next, we used 33 different kinds of cancer expression data to identify the top 200 genes associated with PKP3 expression using GEPIA2. According to Figure 10(b), PKP3 expression is positively correlated with FAM83A (family with sequence similarity 83 member A, *R* = 0.56) and FAM83G (family with sequence similarity 83 member G, *R* = 0.74) genes. There was also a favorable correlation between the aforementioned 5 genes and cancer kinds such as BLCA, ESCA, HNSC, SKCM, Stad, THYM, and PKP3 in the most comprehensive cancer types (Figure 10(c)). To perform KEGG pathway enrichment analysis, we merged these two sets of data. In Figure 11, it appears that “arrhythmic right ventricle cardiomyopathy” and cell adhesion molecules may be implicated in tumor development, suggesting that PKP3 may be involved.

## 4. Discussion

This research revealed that the PKP3 protein structure is highly conserved among different species, based on the gene homology series comparison data. Furthermore, the PKP3 protein is highly conserved in the biological evolution process, according to phylogenetic tree analysis data. Due to the great degree of similarity between the protein sequences, PKP3's normal physiological role may be due to a comparable mechanism. However, whether PKP3 can play a role in the pathogenesis of various cancers through shared molecular pathways has yet to be determined. Previous studies have examined the functional connection between PKP3 and clinical disorders, notably tumors. As big data networks have become more prominent in recent years, researchers have been able to explore this topic by sharing information and performing pan-cancer analyses. Because of this, we used a combination of TCGA, CPTAC, and GEO datasets to examine PKP3's expression pattern, genetic changes, DNA methylation level, and protein phosphorylation sites. 33 distinct cancers were studied in depth and methodically to determine the biological role of the PKP3 gene. Relationships between PKP3 levels and stage, sex, age, body weight, and the presence or absence of the TP53 mutant have been demonstrated for the first time using diverse kinds of tissue from BLCA studies. Data of PKP3-binding proteins and PKP3-associated genes in all cancers were utilized for gene enrichment analysis. There was no statistically significant association between PKP3 expression and Treg cell and T follicular helper cell invasion when several immunological deconvolutions were used. Cancers and normal tissues with BLCA showed decreased DNA methylation in the PKP3 gene promoter and nonpromoter regions. PKP3 DNA methylation may have a role in BLCA carcinogenesis, although further data are needed. The variations in PKP3 DNA methylation in other cancers were not statistically significant, and further data are needed to corroborate these phenomena.

RETRACTED

It has also been shown that breast cancer, clear cell renal cell carcinoma, and lung adenocarcinoma, as well as endometrial carcinoma in the uterus, have different expression levels of total protein, as well as total protein that has been phosphorylated. On the contrary, primary tumors had greater levels of PKP3's total protein expression and its phosphorylation levels on ARM repeat domain amino acid residues N138 and A145 as well as R211 and G329. There is still a chance that high PKP3 phosphorylation by-products offer signals of little practical relevance to tumor cells, and further investigations are needed to examine the possible function of high PKP3 phosphorylation in tumorigenesis-related regulation. Reduced overall survival prognosis was statistically linked with high PKP3 expression in numerous cancers such as CESC and KIRH as well as MESO, PAAD, and SKCM. The disease-free survival (DFS) study showed that decreased expression of PKP3 was negatively linked with improved prognosis in TCGA instances of KIRC, MESO, PAAD, and PRAD. There are two important reasons to analyze the discrepancies between these two assessments. There are a few reasons for this, including the fact that the statistics are different and that the new survival information may not be picked up by the database. Also, various data processing algorithms are at fault. Our analytical results will be skewed for all of the reasons listed above. A study of the LIHC tumor's Cox regression survival data was done utilizing the OncoLnc Web server (http://www.oncolnc.org/); however, the results were unremarkable. To establish the significance of PKP3 in survival and prognosis in patients with different kinds of cancer, further research will require bigger clinical samples. Studies have demonstrated that PKP3 regulates cadherin binding, which is crucial for cell-cell adhesion. Based on the Kaplan–Meier mapping dataset containing GEO data, we also observed a positive correlation between PKP3 expression and cell adhesion molecules.

RETRACTED

## 5. Conclusion

Except for hepatocytes and cardiomyocytes, PKP3, the most extensively expressed member of the PKP family, is found in monolayer and stratified epithelial tissues containing desmosomes. It is sufficient to demonstrate that PKP3 plays an important role in the prognostic evaluation and is a possible therapeutic target for ovarian cancer. In this paper, we further examined PKP3 expression, genetic methylation, and protein phosphorylation. These are all associated with clinical prognosis, according to this first pan-cancer study of PKP3. Additionally, we found that PKP3 expression can alter the microenvironment of tumor cells by causing immune cells to infiltrate the tumor cells. For the first time, PKP3's involvement in malignancies has been comprehensively examined by this work.

In the future, we want to offer an approach that automatically optimizes the framework's configuration parameters utilizing gene expression programming and the particle swarm optimization technique. This would significantly improve the suggested model's performance in terms of computation speedup.

## Figures and Tables

**Figure 1:** Proposed model architecture.

**Figure 2:** Expression analysis of PKP3 gene in different tumors.

**Figure 3:** Expression analysis of PKP3 protein in different pathological stages.

**Figure 4:** Expression of PKP3 is linked to prognosis in tumors.

**Figure 5:** Mutational characteristics of PKP3 in different TCGA tumors.

**Figure 6:** Mutation PKP3 was associated with clinical survival prognosis in different cancers.

**Figure 7:** Analysis of PKP3 DNA methylation level.

**Figure 8:** Promoter methylation level analysis of PKP3 in the BLCA tumors.

**Figure 9:** Phosphorylation analysis of PKP3 protein in different tumors.

**Figure 10:** The correlation between PKP3 expression and immune cell infiltration.

**Figure 11:** Enrichment analysis of PKP3-related genes.

## Data Availability

The datasets used and/or analyzed during the current study are available from the corresponding author on reasonable request.

## Supplementary Materials

Supplementary Materials Figure S1: structural characteristics of PKP3 in different species. Figure S2: phylogenetic tree of PKP3. Figure S3: the expression level of PKP3 in different organs and tissues under normal physiological conditions. Figure S4: the expression level of PKP3 in different tumors. Figure S5: the expression level of PKP3 in different pathological stages of tumor. Figure S6: analysis of the correlation between PKP3 expression and tumor survival prognosis. Figure S7: correlation between PKP3 gene expression and prognosis of cancers using the Kaplan–Meier plotter. Figure S8: correlation analysis between PKP3 expression and infiltration of immune cells.

RETRACTED

## References

[1] Belli C., Trapani D., Viale G. (2018). Targeting the microenvironment in solid tumors. *Cancer Treatment Reviews*.

[2] Walsh C. J., Hu P., Batt J., Dos Santos C. C. (2016). Discovering MicroRNA-regulatory modules in multi-dimensional cancer genomic data: a survey of computational methods. *Cancer Informatics*.

[3] Hongzhen Z., Yanyu L., Xuexiang L. (2019). The diagnostic and prognostic significance of long non-coding RNA CRNDE in pan-cancer based on TCGA, GEO and comprehensive meta-analysis. *Pathology, Research & Practice*.

[4] Pei J., Zhong K., Li J., Xu J., Wang X. (2021). ECNN: evaluating a cluster-neural network model for city innovation capability. *Neural Computing & Applications*.

[5] Yang X., Shao X., Gao L., Zhang S. (2016). Comparative DNA methylation analysis to decipher common and cell type-specific patterns among multiple cell types. *Briefings in functional genomics*.

[6] Broussard J. A., Getsios S., Green K. J. (2015). Desmosome regulation and signaling in disease. *Cell and Tissue Research*.

[7] Fischer-Keso R., Breuninger S., Hofmann S. (2014). Plakophilins 1 and 3 bind to FXR1 and thereby influence the mRNA stability of desmosomal proteins. *Molecular and Cellular Biology*.

[8] Hatzfeld M., Wolf A., Keil R. (2014). Plakophilins in desmosomal adhesion and signaling. *Cell Communication and Adhesion*.

[9] Lim V., Zhu H., Diao S., Hu L., Hu J. (2019). PKP3 interactions with MAPK-JNK-ERK1/2-mTOR pathway regulates autophagy and invasion in ovarian cancer. *Biochemical and Biophysical Research Communications*.

[10] McCrea P. D., Gottardi C. J. (2016). Beyond *β*-catenin: prospects for a larger catenin network in the nucleus. *Nature Reviews Molecular Cell Biology*.

[11] Schmidt A., Langbein L., Prätzel S., Rode M., Rackwitz H.-R., Franke W. W. (1999). Plakophilin 3-a novel cell-type-specific desmosomal plaque protein. *Differentiation*.

[12] Demirag G. G., Sullu Y., Yucel I. (2012). Expression of Plakophilins (PKP1, PKP2, and PKP3) in breast cancers. *Medical Oncology*.

[13] Ishiyama N., Ikura M. (2012). The three-dimensional structure of the cadherin-catenin complex. *Subcellular Biochemistry*.

[14] Chandrashekar D. S., Bashel B., Balasubramanya S. A. H. (2017). UALCAN: a portal for facilitating tumor subgroup gene expression and survival analyses. *Neoplasia*.

[15] Kundu S. T., Gosavi P., Khapare N. (2008). Plakophilin3 downregulation leads to a decrease in cell adhesion and promotes metastasis. *International Journal of Cancer*.

[16] McMillan J. R., Akiyama M., Shimizu H. (2003). Alterations in desmosome size and number coincide with the loss of keratinocyte cohesion in skin with homozygous and heterozygous defects in the desmosomal protein plakophilin 1. *Journal of Investigative Dermatology*.

RETRACTED

[17] Sobolik-Delmaire T., Katafiasz D., Keim S. A., Mahoney M. G., Wahl J. K. (2007). Decreased plakophilin-1 expression promotes increased motility in head and neck squamous cell carcinoma cells. *Cell Communication and Adhesion*.

[18] Hofmann I. (2020). Plakophilins and their roles in diseased states. *Cell and Tissue Research*.

[19] Sklyarova T., Bonné S., D’Hooge P. (2008). Plakophilin-3-deficient mice develop hair coat abnormalities and are prone to cutaneous inflammation. *Journal of Investigative Dermatology*.

[20] Chen Z., Yu M., Guo L. (2020). Tumor derived SIGLEC family genes may play roles in tumor genesis, progression, and immune microenvironment regulation. *Frontiers in Oncology*.

[21] Li B., Severson E., Pignon J.-C. (2016). Comprehensive analyses of tumor immunity: implications for cancer immunotherapy. *Genome Biology*.

[22] Li T., Fan J., Wang B. (2017). TIMER: a web server for comprehensive analysis of tumor-infiltrating immune cells. *Cancer Research*.

[23] Guo L., Li X., Liu R., Chen Y., Ren C., Du S. (2020). TOX correlates with prognosis, immune infiltration, and T cells exhaustion in lung adenocarcinoma. *Cancer Medicine*.

[24] Tang Z., Kang B., Li C., Chen T., Zhang Z. (2019). GEPIA2: an enhanced web server for large-scale expression profiling and interactive analysis. *Nucleic Acids Research*.

[25] Chen F., Chandrashekar D. S., Varambally S., Creighton C. J. (2019). Pan-cancer molecular subtypes revealed by mass-spectrometry-based proteomic characterization of more than 500 human cancers. *Nature Communications*.

[26] Lin W., Wu S., Chen X. (2020). Characterization of hypoxia signature to evaluate the tumor immune microenvironment and predict prognosis in glioma groups. *Frontiers in Oncology*.

[27] Zhang Q., Huang R., Hu H. (2020). Integrative analysis of hypoxia-associated signature in pan-cancer. *iScience*.

[28] Zhang Z., Lin E., Zhuang H. (2020). Construction of a novel gene-based model for prognosis prediction of clear cell renal cell carcinoma. *Cancer Cell International*.

[29] Cerami E., Gao J., Dogrusoz U. (2012). The cBio cancer genomics portal: an open platform for exploring multidimensional cancer genomics data: figure 1. *Cancer Discovery*.

[30] Gao J., Aksoy B. A., Dogrusoz U. (2013). Integrative analysis of complex cancer genomics and clinical profiles using the cBioPortal. *Science Signaling*.

[31] Unberath P., Knell C., Prokosch H. U., Christoph J. (2019). Developing new analysis functions for a translational research platform: extending the cbioportal for cancer genomics. *Studies in Health Technology and Informatics*.

RETRACTED

[32] Wu P., Heins Z. J., Muller J. T. (2019). Integration and analysis of CPTAC proteomics data in the context of cancer genomics in the cbioportal. *Molecular & Cellular Proteomics*.

[33] Morris T. P., Jarvis C. I., Cragg W., Phillips P. P. J., Choodari-Oskooei B., Sydes M. R. (2019). Proposals on Kaplan-Meier plots in medical research and a survey of stakeholder views: KMunicate. *BMJ Open*.

[34] Aran D., Hu Z., Butte A. J. (2017). xCell: digitally portraying the tissue cellular heterogeneity landscape. *Genome Biology*.

[35] Aeschbach R., Löliger J., Scott B. C. (1994). Antioxidant actions of thymol, carvacrol, 6-gingerol, zingerone and hydroxytyrosol. *Food and Chemical Toxicology*.

[36] Szklarczyk D., Gable A. L., Lyon D. (2019). STRING v11: protein-protein association networks with increased coverage, supporting functional discovery in genome-wide experimental datasets. *Nucleic Acids Research*.

